# Phytochemical and GC-MS analysis of *Thevetia peruviana* fruit methanol extract as an anti-rodenticide potential against balb C rats

This article has been retracted.

**DOI:** 10.1016/j.heliyon.2024.e29012

**Published:** 2024-04-02

**Authors:** Anthony Irungu Ndung'u, Joseph Mungai Keriko, Patrick Gachoki Kareru, Sammy Indire Wanakai, George Kiprono Kisoi, Grace Gakii Keddy

**Affiliations:** a Chemistry Department, Jomo Kenyatta University of Agriculture and Technology, P. O BOX 62,000-00200, Nairobi, Kenya; b Department of Biochemistry, Jomo Kenyatta University of Agriculture and Technology, P. O BOX 62,000-00200, Nairobi, Kenya; c Department of Chemistry, Catholic University of Eastern Africa, P. O BOX 62157-00200, Nairobi, Kenya

**Keywords:** GC-MS, *Thevetia peruviana*, Secondary metabolites, Anti-rodenticide

## Abstract

Rodents have remained a menace to humans, hence there is need to evaluate for anti-rodent activity of cheap and environment friendly control methods. This study aimed at evaluating the anti-rodenticidal activity of *Thevetia (T.) peruviana* fruit methanol extract. *T. peruviana* fruit was sampled, dried and extracted using methanol/water in the ratio of 3:1 by volume. Phytochemicals; alkaloids, phenols, flavonoids, glycosides, saponins, and tannins were determined qualitatively and quantitatively in the fruit extract. The extract was then characterized using Fourier Transform Infrared (FTIR) and Gas Chromatography Mass Spectrophotometer (GC-MS). Anti-rodent activity of the extracts was determined on a total of 25 mice with body weights of 20–25 g. The animals 8–12 weeks' old were grouped into 5 cages (5 animals per cage), marked and allowed to acclimatize with laboratory conditions of 25 °C, warm or less humid for 5 days with enough water and food. Extract dose (between 0.3 and 0.5 g of extract/kg body weight) was then administered in a single dose by gavage using intubation canula for 7 days and the animals observed for any toxicity and mortality. The data was subjected to probit analysis and ANOVA. Phytochemical screening showed that the extracts contained glycosides, phenols, saponins, alkaloids, triterpenoids, and flavonoids in different abundance. *T. peruviana* fruit contained 125.13 ± 1.04 mg/g in GAE phenolic content, 85.70 mg/g in RE of dry weight of flavonoids, 10.50 ± 0.01 mg/g in TAE of Tannins, 16.50± 0.21 mg/g alkaloid content, and 8.28± 0.11 mg/g saponin content. The FTIR spectrophotometer depicted O – H, CH_2_, C=O, C–O–C functional groups in wave numbers of 3335, 2932, 1599, and 1001 cm^−1^ respectively. The *T. peruviana* fruit methanol extracts depicted high acute toxicity with an average of 300 mg/kg upon oral administration in Balb C mice species. The fruit extract from *T. peruviana* revealed presence of alkaloids, phenols, glycosides, saponins, tannins. These participated synergistically in killing the rats and the postmortem examination report indicated that the tested extract induced a number of physical changes in the mice and therefore the *T. peruviana*'s fruit extract can be utilized as a natural alternative anti-rodent in agriculture production before and after harvesting.

## 1 Introduction

Plants are rich in tremendous amount of bioactive molecules such as terpenoids, alkaloids, flavonoids, glycosides, carbohydrates, etc. which have been found to have biological activities such as antioxidant, antimicrobial and toxicity effect [1]. Yellow (Y.) oleander (*T. peruviana*) is a well-known poisonous shrub grown in gardens and public areas and contains numerous toxic compounds. It is one of the evergreen plant of oleander family that belongs to the Apocynaceae family and is found in the tropical America and Africa, while other species of these family are the *Nerium oleander* from Mediterranean basin and Asia (Fig. 1) [[2], [3], [4]]. It is a shrubby and ornamental tree that grows to about 4.5 m high with pointed leaves of about 5 cm long 0.5 cm wide sub obtuse, acute at base, coriaceous dark green glossy on top, paler underneath leaf and spirally configured. It has yellow flowers and the fruits are juicy black which first grow green and then become black on ripening and the fruit longitudinally divided cream colored which can be utilized through solvent extraction to form biodiesel [[5], [6], [7], [8]]. These fruits are triangular in shape with a fleshy mesocarp and green epicarp, which turns black when ripe. Toxicity has been reported to extend to the latex of the plant which causes a variety of reactions and allergies from irritation to acute respiratory failure. Active compounds in toxicity reported are the glycosides of the cardinalin type which cause poisoning [[5], [6], [7]].

**Fig. 1:** *T. peruviana* tree with yellow flowers. (For interpretation of the references to color in this figure legend, the reader is referred to the Web version of this article.)

Knowledge about the toxicity of *T. peruviana* has been clear since ancient times, with fatal poisoning of insects, animals, and humans. Generally, all parts of the plant are highly toxic because of the presence of contents of cardiac glycosides; a number of components such as Thevetin and Thevetoxin [3,9,10]. Thevetin, a compound contained in a milky sap called Latex is reported present in entirely the whole plant and is employed as a heart stimulant but is extremely poisonous. Other components include Neriifolin, Peruvoside, Ruvoside and Thevetoxin which release gastric and cardio toxic effects [5]. Rupesh et al., and Shieunda & Keriko reported the presence of carbohydrates, proteins, amino acids, fatty oils, alkaloids, glycosides, flavonoids, and volatile oils which they showed that the plant has pharmacognostial potential [11,12].

*T. peruviana* seed extract has been reported to have antimicrobial activity [1], as human food for nutritional supplementation [11], the fruit extract has wound heling ability [13], and anti-termite activity [14]. For instance, the antimicrobial activity of in vitro callus and plant cell suspension cultures of *T. peruviana* extracts was evaluated by disk diffusion tests against gram negative (*Salmonella thipimurium* and *Escherichia coli*) and gram positive (*Staphylococcus aureus* and *Bacillus cereus*) strains of which methanol and ethanol extracts showed considerable antimicrobial activity against these strains [4]. With the contents of glycosides present in *T. peruviana,* the plant has been reported to have toxicity effected and when an extract from any part of the *T. peruviana* plant is ingested, it results to clinical symptoms such as diarrhea, vomiting, nausea, dysrhythmias, restlessness, and abdominal pain [10]. Toxicity of *T. peruviana* has been related to digitalis toxicity where pathophysiology involves direct inhibition of sodium ion (Na^+^) – potassium ion (K^+^) – ATpase pump of the heart and increased vagal gone through increase of intercellular concentrations of Ca^2+^ and Na ^+^ [2,5].

Rodents destroy crops by reducing the overall crop yield and increasing pest control costs. This therefore, reduces crop production and could effectively have significant total economic impacts [[15], [16], [17], [18]]. In agriculture, post-harvest losses occur after harvest if no interventions are made with major loses from insects, pathogens, and rodents [16]. Various synthetic products used for rat control have been employed in trapping and killing rats of which most of them have heavy metals such as zinc and arsenic which contribute to environmental pollution and are highly toxic. These products referred to as rodenticides are synthetic chemical-based rodenticides are widely used and widely available. Rodenticides are pesticides that are chemically designed to kill rodents. They primarily target mice and rats; however, rodenticides can poison animals other than mice and rats. Unintentional rodenticide exposure can have serious consequences for virtually any animal, including birds and humans [19]. Most rodenticides are toxic when consumed, inhaled, or come into contact with the skin as a contact or food toxicant, and the clinical manifestations caused by these rodenticides are severe. Traditional synthetic rodenticides are formulated as baits that are appealing to animals rather than rodents. Therefore, there is need to find green and safe ways of preventing destruction caused by rodents. Natural products have been employed in agriculture in controlling pests as biocontrol agents and are becoming more popular and are being considered as viable replacement methods for controlling various plant diseases because the environment is safer and, in some cases, the only option for protecting plants against pathogens. Besides, these plants have solved the pathogen-resistant breed development which has become a worldwide problem, and most farmers' have shifted their attitudes toward the use of pesticides for crop protection and crop production [20]. Plants have fiber [21] and other phyto-compounds which play a big role as they have antioxidant ability and antimicrobial activity. As we employ fiber in reinforcement of materials, it is important to find use of plants in pesticides applications [21]. The toxicity effect reported in *T. peruviana* leaf, root and fruit extract has not yet been fully exploited as an anti-rodenticide and this study aimed at exploiting the toxicity of *T. peruviana* fruit in developing an anti-rodent [19,22,23].

The aim of this study was to evaluate the toxic effects of methanol/water extract of *T. peruviana* fruit and histopathological changes in the heart, liver, and kidney of albino rats to evaluate the anti-rodenticidal ability. *T. peruviana* extract was orally administered after extraction on the same day at doses of 1 mL and 2 mL of the extract/kg of body weight in 0.5 mL of saline. The results showed that the extract had considerable pathological changes which were perceived in the heart, kidney and liver tissue. Besides, the animals died after a number of days hence, it can be concluded that exposure to *T. peruviana* fruit extract adversely affects the heart, kidney and liver thus being fatal and can be used as an anti-rodent.

## 2 Materials and methods

### 2.1 Materials/requirements

Chemicals: 99.8 % Methanol, Gallic Acid, 5 % sodium nitrite, 1 N Folin-Ciocalteu reagent, 0.1 mM DPPH solution, 10 % aluminium chloride, tannic acid, Mayer reagent, 5 % sodium carbonate, Lead acetate, Ferric chloride, 4 % sodium hydroxide, Alkaline reagent, Iodine solution, sodium hydroxide, Wagner's reagent, and Molisch's reagent.

### 2.2 Sample collection and pre-treatment

*T. peruviana* fruits were collected from Jomo Kenyatta University of Agriculture and Technology Botanical Garden, Kiambu County, Kenya at GPS code Latitude 1° 5′ 35“S, Longitude 37° 0′ 43″ E, after being authenticated by a taxonomist in the month of May 2021. The samples were then transported in plastic bags to the JKUAT GK Botany Laboratory. The voucher specimens were deposited (in triplicates) at JKUAT Botany Herbarium and given accessory voucher numbers AIN–JKUATBH/001/2021. The fruits were selected and thoroughly washed with running tap water to remove dusts and other unwanted materials and cut into small pieces for air drying under shade on the Laboratory benches at room temperature for ten days. The dry samples were then ground into fine powder, weighed, packed and stored in clean dry plastic bags.

### 2.3 Extraction

Extraction involved the method employed by Ngugi et al. (Ngugi et al., 2017), with modifications. Briefly, the ground powder 300 g was weighed into a 2 L conical flask and soaked in methanol – water (3:1) solution. The mixture was placed in a mechanical shaker model for 3 h at 130 RPM, and allowed to stand for three days. The extract was then filtered in a Whatman No. 1 filter paper and concentrated using a rotary evaporator at 45 °C to obtain a solid extract which was weighed and percentage yield calculated.

### 2.4 Phytochemical analysis

#### 2.4.1 Detection of phenolic compounds

Was performed using the Lead acetate test by weighing 50 mg of methanol extract dissolving in distilled water and adding 3 mL of 10 % lead acetate solution. The presence of phenolic compounds was indicated by a bulky white precipitate.

#### 2.4.2 Detection of flavonoids

Was performed using the alkaline reagent test. An aqueous solution of the extract was treated with 10 % ammonium hydroxide solution. Yellow fluorescence indicated the presence of flavonoids.

#### 2.4.3 Detection of saponins

Saponins were detected using the Frothing test. 50 mg of extract was diluted with distilled water to make up to 20 mL. The suspension was shaken for 15 min. A 2-cm layer of foam indicated the presence of saponins.

#### 2.4.4 Detection of alkaloids

Hager's test was used to detect for Alkaloids. 50 mg of solvent-free extract was diluted with few mL of dilute hydrochloric acid and filtered. 2 mL Hager's reagent (saturated aqueous solution of picric acid) was added to a few mL of the filtrate. A prominent yellow precipitate indicated presence of alkaloids.

### 2.5 Quantitative analysis

Qualitative analysis of the phenols, flavonoids, alkaloids, saponins, and tannins was performed using a method described by Ref. [24].

#### 2.5.1 Total phenolic content

Working standard solutions of concentrations of 2.5, 5.0, 7.5, 10.0, and 12.5 μg/mL 50 μL of the standardcts containing phenols were prepared and analysis performed in triplicates, and the contents of all the test tubes were made up to 1 mL with distilled water. Three test tubes marked ‘B’ with 1 mL of distilled water served as the blank and other three test tubes marked P with 100 μL extract each of 0.1 mg sample in 1 mL methanol. 0.5 mL Folin-Ciocalteu (1 N) was then added to each test tube including the blank, test tubes vortexed and allowed to stand for 5 min at room temperature. 2.5 mL of 5 % sodium carbonate was added to all the test tubes including the blank, test tubes vortex and incubated in the dark at room temperature for 40 min. The absorbance of the blue color developed against the reagent blank at 725 nm was measured using spectrophotometer. The amount of total phenol content in the sample was calculated using equation (1) below and expressed as mg/g of the Gallic acid Equivalent [25].

(1) $$C=c_{1\;}x\;\frac{V}{m}$$

Where *C* = total phenolic content in mg/g, in GAE (Gallic acid equivalent), c_*1*_ = concentration of the Gallic acid established from the calibration curve in mg/mL, *V* = volume of extract in mL. and *m* = the weight of the plant extract in g.

#### 2.5.2 Total tannins content

100 mg of Polyvinyl polypyrrolidone (PVPP) was weighed in 2 mL Eppendorf tubes. 500 μL of plant sample and 500 μL of distilled water was added. The tubes were incubated for 4 h at 4 °C. The Eppendorf tubes were centrifuged at 3000 rpm for 10 min at 4 °C after incubation. The supernatant contained only the non-tannin phenolic. Working standard solution concentrations were prepared as shown in the phenols100 μL of non-tannin phenolic extract of sample (in triplicates) was added into series of test tubes, and the contents of all the test tubes was made up to 1 mL with distilled water. The test tube marked ‘B’ with 1 mL of distilled water served as the blank. 0.5 mL Folin-Ciocalteu reagent (1 N) was added to each test tube including the blank, t vortexed and allowed to stand for 5 min at room temperature. 2.5 mL of 5% sodium carbonate was added to all the test tubes including the blank, the test tubes vortexed and incubated in the dark at room temperature for 40 min. The absorbance of the blue color developed against the reagent blank at 725 nm was measured using spectrophotometer. The amount of tannins in the sample was calculated using equation (2) below and expressed as mg/g of the Tannic Acid Equivalent [25].

(2) $$C=c_{1\;}x\;\frac{V}{m}$$

Where *C* = total tannin content in mg/g, in TAE (Tannic acid equivalent), *c*_*1*_ = concentration of the Tannic acid established from the calibration curve in mg/mL, *V* = volume of extract in mL. and *m* = the weight of the plant extract in g.

#### 2.5.3 Flavonoid content

W working standard solutions of concentrations 8, 16, 24, 32, and 40 μg/mL concentrations, respectively and 50 μL of extract of sample were taken into series of test tubes and the analysis performed in triplicates. The contents of all test tubes were made up to 1 mL with distilled water with test tube marked ‘B’ with 1 mL of distilled water served as the blank. 150 μL of 5 % sodium nitrite was then added to each test tube, the test tubes vortexed and incubated at room temperature for 5 min. Then 150 μL of 10 % aluminium chloride was added to all test tubes vortexed again and incubated at room temperature for 6 min 2 mL of 4% sodium hydroxide was added and the contents of test tubes made up to 5 mL using distilled water. The test tubes were vortexed and allowed to stand for 15 min at room temperature. The absorbance of the pink color developed due to the presence of flavonoids against the reagent blank at 510 nm was measured using the spectrophotometer. The amount of flavonoids in the sample was calculated using equation (3) below and expressed as mg/g of the Rutin acid Equivalent [25].

(3) $$C=c_{1\;}x\;\frac{V}{m}$$

Where *C* = total flavonoid content in mg/g, in RAE (Rutin acid equivalent), *c*_*1*_ is the concentration of the Rutin acid established from the calibration curve in mg/mL, *V* is the volume of extract in mL. and *m* is the weight of the plant extract in g.

### 2.6 Characterization of the extract

#### 2.6.1 Fourier Transform Infrared

The Shimadzu Fourier Transform Infrared spectrophotometer (FT-IR) (FTS- 8000, Japan) was used to analyze functional groups present on the plant extract by the standard KBr method, with spectral resolution set at 4 cm^−1^ and the scanning range from 400 to 4000 cm^−1^. The samples were ground with KBr in the ratio of 1 mg–10 mg in a mortar and pestle, and 1 mg of homogenous mixture placed in sample discs pressed using a hydraulic press and mounted into the FT-IR machine for analysis [26].

#### 2.6.2 Gas chromatography Mass Spectrophotometer (GC–MS)

To remove interfering matrices, the samples were first cleaned up using sample cleanup procedure, the analyte concentrated and the sample matrix changed to GC grade before analysis. Briefly, the solid phase extraction procedure employed C_18_ cartilage conditioned with 3 mL of methanol then 3 mL of sample was loaded to allow it flow slowly out of the cartilage giving it enough time to interact with adsorbent. The sample was then allowed to dry in a stream of air for 10 min and thereafter eluted with 3 mL methanol into a 4 mL vial, concentrated using genetic concentrator, reconstituted with 1 mL of methanol, filtered using nylon micro filters size 0.22 μM into 1.5 mL vials and taken to GC-MS for analysis. GC–MS analysis of crude *T. peruviana* was evaluated using a shimadzu GC–MS at JKUAT, Analytical laboratory. 5 g of the powdered plant samples was extracted with Acetonitrile, then solvent exchanged with 2, 2, 4-Trimethylpentane before GCMS analysis. GC–MS technique was used for identification of the chemical compounds present in the extracts and it was carried out on Agilent 5975 GC–MS operating in EI mode at 70 eV with a mass range of 40–400 *m*/*z*. A capillary column 30 m × 0.25 mm (id) and Helium gas was used as carrier gas with flow rate of 1.2 mL/min and oven temperature of 60 °C [27].

### 2.7 Animals and experimental design

#### 2.7.1 Handling of animals

Adult males and females balb C rats were used for experiments. A total of 25 male mice with body weights of 20–25 g were purchased from the Laboratory of Small Animal Facility for Research and Innovation (SAFARI) at Jomo Kenyatta University of Agriculture Technology, Kenya. The mice were housed in cages (5 mice per cage) in a well ventilated room with enough light and temperature (20–25 °C). Food and water was availed for the animals. The animal management protocol and the experimental design was accepted by the Research Ethics Committee, Jomo Kenyatta University of Agriculture Technology, Kenya [28].

#### 2.7.2 Acute oral toxicity test

Acute oral toxicity of *T. peruviana* methanol extract was performed using a previous work done with modifications [16,29]. In brief, the test principle based on a stepwise method with use of a minimum number of animals per step. Balb C mice were randomly selected, marked to allow individual identification, and kept in cages for 5 days before dosing to allow for acclimatization to the Laboratory conditions. The extract dose was prepared shortly prior to administration. The *T. peruviana* methanol fruit extract dose was administered in a single dose by free choice feeding test which was important to determine the palatability of the extract on food offered [28]. The dosage offered had 0.5 g of dried extract/kg body weight after reconstitution in 0.5 mL of saline. The extract was employed using a stepwise procedure, each step using five animals of both sex (females and males). Female balb C mice used were nulliparous and non - pregnant. Each mouse, at the commencement of its dosing, was between 8 and 12 weeks old and doses between 0.5 and 3.0 g of dried extract/kg body weight were used after reconstitution in 0.5 mL of saline and administered orally by stomach gavage for 7 days [16,29]. 24 hr observation of the animals’ apparent signs of toxicity and mortality was performed according to method employed previously [29,30].

### 2.8 Histopathology

Histological studies were performed in JKUAT histology laboratory. The liver was placed in 10 % formalin, dehydrated in increasing series of ethanol, cleared in xylene and inserted in paraffin. Sections of 6 μm thickness from the control and the test were cut out, stained with hematoxylin, and eosin stain, and examined using a light microscope. The heart muscles were washed with normal saline solution (0.9 % NaCl in distilled water) and then fixed in 10 % buffered formalin. After standard processing of the tissue, 5 μm sections were prepared and stained with hematoxylin and eosin. The slides were then examined under a light microscope at a magnification of ×1000 to investigate the histopathological changes. All images were captured with a calibrated standard digital microscope camera (IVU5100 digital microscope, Labomed America Incl. USA) for image capture and enhancement. A semi-quantitative microscopy system for myocardial damage was applied based on the severity and extent of the lesions observed in each mouse. Briefly, for each myocardial slide, histopathological signs of inflammation and/or myocarditis were seen.

### 2.9 Data analysis

The data was subjected to probit analysis and ANOVA.

## 3 Results and discussion

### 3.1 Phytochemical analysis

The use of plant extracts as pesticides depends on knowing their chemical constituents, hence, it is important to carry out preliminary phytochemical screening for extracts of *T. peruviana* fruit.

Table 1 shows the summarized phytochemical screening of chemical constituents of guava leaf extracts under study on qualitative basis.

**Table 1:** Phytochemical screening.

Test	Observation
Tannins	+
Phenols	+
Flavonoids	+
Alkaloids	+
Saponins glycosides	+

Key: + presence of constituents; - absence of constituents.

The phytochemical screening of chemical constituents of *T. peruviana* fruit extract revealed the presence of active compounds; phenols, saponins, tannins, flavonoids, and alkaloids which are known to exhibit medicinal and physiological activities. For instance, tannins are polyphenolic compounds that bind to proline rich protein that interferes with protein synthesis and has known to have antibacterial activity. Flavonoids are hydroxylated polyphenolic compounds produced by plants in response to microbial infections to which this aspect has been extensively studied and found to have antimicrobial activity against an array of microorganisms in vitro [5,31]. Also they have a capacity to act as an antioxidant; it has been reported that the flavones and catechins seem to be the most powerful flavonoids for protecting the body against reactive oxygen species [28]. These molecules are toxic and cause poisoning to mammals [2].

### 3.2 Total flavonoid, phenolic, tannins, alkaloids and saponnin contents

The total flavonoid, phenolic, tannins were obtained using the spectrophotometric method while alkaloids and saponin contents were done using gravimetric method. Fig. 2 below shows the standard calibration curves for phenolics, flavonoids, and tannins, respectively.

**Fig. 2:** Standard graphs of A (Phenols), B (Flavonoids) and C (Tannins).

Graphs in Fig. 2 above were drawn for the phenolic, flavonoids and tannins standards; gallic, rutin and tannic acids, respectively. The graphs were used to analyze the concentrations of phenolics, flavonoids and tannins in the dry plant samples and reported as garlic acid equivalents (GAE)/g of dry weight extract (DW), mg of Rutin equivalent (RE)/g of dry weight of sample, and mg of Tannic acid equivalent (TAE)/g of dry weight of sample and results are as shown in Table 2 below. Table 2 shows the total phenolic, flavonoids and tannins content of *T. peruviana* extracts.

**Table 2:** Total Phenolic, Flavonoids, Alkaloids, Saponins, and Tannins Content in *T. peruviana* (*T. peruviana*) fruit extracts.

Secondary Metabolites	*T. peruviana* Methanol Fruit Extract
Phenols (mg/g in GAE of Dry Weight)	125.13 ± 1.04
Flavonoids (mg/g in RAE of Dry Weight)	85.70 ± 0.17
Alkaloids mg/g of Dry Weight	16.50 ± 0.21
Saponins mg/g of Dry Weight	14.53 ± 0.12
Tannins (mg/g in TAE of Dry Weight)	10.50 ± 0.01

From the data (Table 2), *T. peruviana* extract contained more polyphenols and flavonoids. Besides, the extract also contained significant amounts of alkaloids, saponins, and tannins. These compounds contain considerable amounts of glycosides attached which provide medicinal value as well as toxic effect.

### 3.3 Fourier Transform Infrared analysis

The FTIR (FTS 8400) located at the Jomo Kenya University of Agriculture and Technology was employed in determination of the functional groups present on the plant extracts (Fig. 3).

**Fig. 3:** FTIR of the *T. peruviana* methanol fruit extract.

From the spectra (Fig. 3), the *T. peruviana* extract exhibited ten distinct peaks. The peak observed at 3335 is due to the OH stretching, CH_2_ stretching 2932 cm^−1^, C=O at 1599, and C–*O*–C ether at 1001 cm^−1^, respectively Table 3.

**Table 3:** Summary of the Functional groups present on *T. peruviana* methanol extract.

Functional Group	Peak	Probable compounds
OH	3334.9	Alkaloids, flavonoids, polyphenol, tannins
C–H	2935.8	Alkaloids, flavonoids, polyphenol, tannins
C=C	1594.2	Alkaloids, flavonoids, polyphenol, tannins
Esters	1114.1	Alkaloids, flavonoids, polyphenol, tannins
C–*O*–C	1070.2	Alkaloids, flavonoids, polyphenol, tannins

The extract exhibited the presence of a broad peak for hydrogen - oxygen bonded –OH stretching in the functional group region. Presence of this functional groups is attributed to the presence of polyphenols, tannins, alkaloids, and flavonoids - containing phytochemicals in the leave extracts of *T. peruviana.* These strong and intense peaks observed confirmed the glycosidic linkage [16,24]. Most studies show that a number of plant metabolites, including polyphenolic substances such as flavonoids and tannins and various herbal extracts, show antioxidant, anti-inflammatory, and antimicrobial activities.

### 3.4 Gas Chromatography-Mass Spectrophotometer (GC-MS) analysis

GC–MS analysis was used to identify the compounds present in the methanol extract of *T. peruviana* and the spectrum below was obtaine (Fig. 4).

**Fig. 4:** GC-MS chromatogram of *T. peruviana* extract.

Secondary metabolites present in *T. peruviana* extract were identified with the help of Gas Chromatography – Mass Spectrophotometer and the results are depicted in Table 4 below.

**Table 4:** Some secondary metabolites identified using GC–MS with the help of a NIST 17 spectral data base.

Compounds present				
RT	RT Compound	MF	MW	Class
5.914	terpineol	C_12_H_17_F_3_O_2_	260	Alcohol
7.791	Alfa-copaene	C_15_H_24_	206	Alcohol
8.727	2-propenoic acid 3-(2-hydroxyphenyl)- (E)	C_9_H_8_O_3_	154	Hydroxycinnamic acid
9.5540	Lycopodan-8-one,5,12-dihydroxy-15-methyl-(5a,15S)-	C_16_H_25_NO_3_		Ketone
11.068	Caryophyllenyl alcohol	C_15_H_26_O	223	Sesquiterpene Alcohol
12.664	Globulol	C_15_H_26_O	223	Sesquiterpene alcohol
15.546	Cubenol	C_15_H_26_O	223	Sesquiterpene Alcohol
17.347	Rotundene	C_15_H_24_	204	Terpene
21.613	Phytol	C_20_H_40_O	296	Acyclic diterpene
40.422	Lupeol	C_30_H_50_O	426	Triterpene

Volatile compounds including the alcohols, esters, amines, ketones, ethers, oxides, aldehydes, amides, phenols, heterocycles, and terpenes were identified in the *T. peruviana* extracts based on the data obtained (Table 3). Phytol is a diterpene alcohol derived from the degradation of chlorophyll, which is used in the synthesis of vitamins, and it has promising antischistosomal properties in vitro and in a mouse model of schistosomiasis mansoni. Lupeol is an anti-cancer and anti-inflammatory dietary triterpene that aids in the stabilization of phospholipid bilayers in plant cell membranes [32].

### 3.5 Determination of LD_50_

The *T. peruviana* extract exhibited high acute toxicity with LD_50_ cut-off of 300 mg/kg body weight.

It was observed that as the concentration of extract increased, the mortality rate increased as shown above (Table 5). This showed that the extract contains active compounds that are toxic and caused death. However, as the concentration increases, death rate also reduces [33].

**Table 5:** The mice mortality for different formulated anti rodent.

Cages	Weight of extract (g)	Weight of pellets (g)	No. of mice used	No. of dead mice after 72 h
**Cage 1 (1.25% extract)**	0.25	5	5	4 (80%)
**Cage 2 (10% extract)**	0.50	5	5	5 (100%)
**Cage 3 (15% extract)**	0.75	5	5	5 (100%)
**Cage 4 (20% extract)**	1.00	5	5	4 (80%)
**Cage 5 (Control)**	0.00	5	5	0%

### 3.6 The postmortem report of the mice

Acute rodenticides are active and with profound effects on the entire body organs and systems which may lead to outcomes such as paralysis, heart, and kidney failure and finally death. Very fast acting acute rodenticides usually develop feeding avoidance in less poisoned rodents. The postmortem of the control and the test mice was performed which showed a number of differences [34].

Fig. 5 below shows the photos of the mice before and after taking *T. peruviana* methanol fruit extracts.

**Fig. 5:** Animals before and after taking the extract.

From the photo (Fig. 5, S1–S5), the mice were active before taking the food with extract. They had clearly laid fur with normal breathing pace. However, after taking the extract, the animals were stressed and the fur looked shaggy and were restless. Besides, the breathing was fast and the animals laid isolated with minimal movement showing the effect of taking *T. peruviana* methanol fruit extracts.

Fig. 6 below shows the photos of the inner parts of the mice before and after taking *T. peruviana* methanol fruit extracts.

**Fig. 6:** Photo of the Inner parts of the mice before and after taking *T. peruviana* methanol fruit extracts.

From Fig. 6 and S10–S14, it was observed that the intestines, the heart and the kidneys were normal for the control-mice that have not taken the extract. However, the heart, intestines and kidneys of the mice that had fed on food containing *T. peruviana* methanol fruit extracts were swollen and had turned black showing reduced oxygen intake. In general, the intestines of the control and before test were observed to have blood stains and full of health. However, after eating the extract, the intestines had turned black with less blood. This showed that the extract had effect on the intestines after injection [16].

Fig. 7 shows the photo-images of the cross section of the liver for the control balb C mouse and balb C mouse after taking the *T. peruviana* fruit methanol extract.

**Fig. 7:** Photomicrographs of the cross sections from the livers of balb C mice: Control, showing a central vein (CV), cords of liver cells separated by blood sinusoids (S) and Kupffer cells (Arrow) Heapatocytes (H). [B]: After treatment with Ricinus extract, displaying congested central vein (CV), degeneration (D) cellular infiltration (Arrow). Liver after treatment with *T. peruviana* fruit methanol extract, H demonstrates hemorrhage in central vein and blood vessels, necrosis (N).

From the photo-microimages, the hepatocytes contained vesicular and central nuclei and were round in shape. The narrow blood sinusoids separated hepatic cords between the Endothelial and Von Kupffer cells (Fig. 7A). mouse liver sections from those given from the *T. peruviana* extract treatment displayed congestion within the central vein, some regions of degeneration, and cell infiltration close to the central vein (Fig. 7B). hemorrhage was also observed in the central vein and blood vessels [35,36].

Fig. 8 below shows a cross section of the kidneys for the control and the mice after taking *T. peruviana* extract.

**Fig. 8:** Cross section the kidney K1 (Control-before taking *T. peruviana* methanol fruit extracts) and K2 (when exposure to *T. peruviana* methanol fruit extracts).

The kidney is responsible for elimination of waste materials from metabolic processes, foreign materials in the body systems, and maintaining homeostasis [35]. From Fig. 8, the kidney for the control was normal with the cells well-formed and with life. However, kidneys of the mice after taking the extract displayed some changes in the form of the cells and also had black blood stains. Besides, the number of cells was less as compared to the control. Generally, degenerative changes seen in the kidney included necrobiosis in the epithelial cell lining of renal tubules, glomerular tuft congestion of the hypertrophied glomeruli. A number of glomeruli are damaged to flattened renal tubules’ epithelial tissue that lead to hemorrhage and rapture of tubular membrane, and further to inflammation. Degeneration also leads to disruption in cellular metabolism causing morphological abnormalities [30,35].

Fig. 9 displays the cross section of the heart of balb C mice before and after taking *T. peruviana* methanol fruit extracts.

**Fig. 9:** Cross section of the heart before and after taking *T. peruviana* methanol fruit extracts.

From Fig. 9, the cell lining of the heart of the mice that had taken the extract had some black spots as compared to the control. This showed the diffusion nature of the extract through the body system. The weight of the heart increase after taking methanol extract. Besides, noticeable darkness of color was observed [30].

### 3.7 Discussion

The major toxic components are the cardiac glycosides oleandrin and nerin. Phytochemical screening of the extract revealed the presence of phenols, flavonoids, glycosides, alkaloids, saponins and tannins. These compounds were well related with the functional groups identified in the Fourier Transform Infrared spectrophotometer. Besides, gas chromatography displayed presence of alcohols, ketones, terpenes, ethers and aldehydes. These compounds show how effective the compounds present in the methanol fruit extract of *T. peruviana.* The aim of our study was to evaluate the toxic effects of methanol *T. peruviana* fruit extract and histopathological changes in the heart, liver, and kidney. *T. peruviana* extract was orally administered after extraction on the same day at doses of 1 mL and 2 mL of the extract/kg of body weight in 0.5 mL of saline. The results showed marked pathological changes were perceived in behavior of the animals and changes in the heart, kidney and liver tissue. *T. peruviana* contains glycosides which have been reported to be poisonous [37,38]. The presence of the –OH functional group in the extract clearly portrays the presence of glycosides and the effective nature in physiological changes of the heart, liver and kidney. Thus, it can be concluded that exposure to *T. peruviana* fruit extract adversely affects the heart, kidney and liver thus being fatal. A semi-quantitative microscopy system for myocardial damage was applied based on the severity and extent of the lesions observed in each mouse. Briefly, for each myocardial slide, histopathological signs of inflammation and/or myocarditis were seen. Due to the high-dosage, the heart muscles showed severe inter-fascicular oedema with dilated congested vessels and severe degenerated myocytes with focal striation loss and focal vacuolar degeneration. The heart muscles also showed focal marked inter-fascicular oedema with dilated congested vessels and severe degenerated myocytes with vacuolation of the muscle. Additionally, myofibrils showed severe striation loss. Bio-pesticide activity of *T. peruviana* is a broad and excellent means of controlling mice on commercial crops and items. The methanol extract of the fruit of *T. peruviana* showed rodenticidal activity against most of the Balb C mice. Use of these fruits in controlling mice is environmental friendly and the provides environmental balance of the soil [39].

## 4 Conclusion

*T. peruviana* was found to contain alkaloids, phenols, flavonoids, saponins, and glycosides. These compounds were confirmed by FT-IR and GC MS. The *T. peruviana* fruit extracts depicted high acute toxicity with LD_50_ of 300 mg/kg upon oral administration in Balb C mice species. The postmortem examination report indicated that the sacrificed mice and the dead mice had induced physiological changes in the liver, spleen, and heart which included necrosis associated with inflammatory cell infiltration in small intestine and damage in oedema and septa. Therefore, the *T. peruviana*'s fruit extract can be utilized as an anti-rodenticide in agriculture production before and after harvesting.

## Data availability statement

Data associated with this study has not been publicly availed in any repository.

The data has been included in the Article/Supplementary Material/Referenced in article.

## CRediT authorship contribution statement

**Anthony Irungu Ndung'u:** Writing – review & editing, Writing – original draft, Visualization, Validation, Supervision, Resources, Project administration, Methodology, Investigation, Formal analysis, Data curation, Conceptualization. **Joseph Keriko Mungai:** Writing – review & editing, Writing – original draft, Visualization, Validation, Supervision, Resources, Project administration, Methodology, Investigation, Formal analysis, Data curation, Conceptualization. **Patrick Gachoki Kareru:** Writing – review & editing, Writing – original draft, Resources, Methodology, Investigation, Funding acquisition, Data curation, Conceptualization. **Sammy Indire Wanakai:** Writing – review & editing, Writing – original draft, Visualization, Validation, Supervision, Software, Resources, Project administration, Methodology, Investigation, Formal analysis, Data curation, Conceptualization. **George Kiprono Kisoi:** Validation, Resources, Methodology, Investigation, Data curation. **Grace Gakii Keddy:** Visualization, Validation, Resources, Methodology, Funding acquisition, Conceptualization.

## Declaration of competing interest

The authors declare that they have no known competing financial interests or personal relationships that could have appeared to influence the work reported in this paper.
